# Correlation between Retinol Binding Protein 4 and CT Perfusion Imaging and Prognosis in Patients with Acute Ischemic Stroke Based on Cell Imaging Data Analysis

**DOI:** 10.1155/2022/3055712

**Published:** 2022-08-08

**Authors:** Chao Liu, Juxian Gu, Yan Yao, Ping Guo, Hongwei Hu

**Affiliations:** ^1^Department of CT Diagnostics, Cangzhou Central Hospital, Hebei, China; ^2^Cangzhou Central Hospital, Hebei, China; ^3^Cangzhou Medical College, Hebei, China

## Abstract

**Objective:**

In order to explore the correlation between the retinol binding protein 4 (RBP4) and prognosis of patients with acute ischemic stroke (AIS), CT perfusion imaging can be used to scan the brain tissue of patients, which can identify abnormal perfusion areas and ischemic penumbra brain tissue, so as to provide a basis for doctors to formulate a reasonable clinical treatment plan.

**Methods:**

200 patients with first-episode acute ischemic stroke were selected from the Department of Neurology of our hospital, including 128 males and 72 females, aged between 32 and 85 years, with an average age of 45 ± 4.3 years. After admission, the patients were tested for xanthol binding protein 4 in time, the patient's demographic data and the basic clinical data were recorded, the degree of brain injury was evaluated, and the short-term outcome was evaluated after treatment.

**Results:**

A total of 200 AIS patients with different degrees of brain injury were included in this study, including 128 males and 78 females, aged between 32 and 85 years, with an average age of 45 ± 4.3 years. Among them, 100 patients used CT perfusion imaging for brain scanning as the observation group, 100 patients used traditional imaging methods as the reference group, and 100 healthy people were included as the blank group. At the same time, the contents of total cholesterol, triacylglycerol, high-density lipoprotein cholesterol, and low-density lipoprotein cholesterol were measured by using an automatic biochemical analyzer. The patients were evaluated in the early stage of treatment and the effect of prognostic intervention was recorded.

**Conclusion:**

The application of CT perfusion imaging in the adjuvant treatment of AIS patients was helpful to identify the abnormal perfusion area and the brain tissue of ischemic penumbra, so as to provide a basis for doctors' follow-up treatment. At the same time, AIS patients with high serum RBP4 level had mild stroke severity, good short-term prognosis, and improved treatment effect, which improved patients' quality of life.

## 1. Introduction

AIS is often called stroke in traditional Chinese medicine. The disease belongs to nervous system disease. Its pathological essence is that the blood circulation of the local brain tissue is not smooth on the basis of atherosclerosis, resulting in cerebral ischemia and hypoxic injury, which threatens the health of the human nervous system. With the improvement of medical treatment, the mortality rate of stroke has decreased, but there are also common secondary sequelae, which affect the self-care ability of patients.

Relevant data show that the formation of AIS is related to daily habits and eating habits, including hypertension, smoking, alcoholism, excessive stress, mental depression, hyperlipidemia, and lack of exercise. These factors affect the incidence rate of cerebrovascular disease and show a high incidence rate and sequelae, which bring a certain economic burden to patients and affect their self-care ability. However, most patients can reduce the risk of AIS through self-regulation and control.

The incidence rate of this disease is higher in middle-aged and elderly people over 50–60 years. The early symptoms of the disease are not obvious. Some patients may have dizziness, intermittent limb numbness, weakness, and other manifestations. Because the symptoms are unknown and the duration is short, they are often ignored by the patients. And the onset of the disease is more urgent. A few hours after the onset is the golden rescue time of the disease, which is related to the prognosis of patients. Different individuals have different prognosis. Early intervention for AIS patients is helpful to control the patient's condition, so as to improve the cure rate and reduce the related sequelae.

In recent years, spiral CT perfusion imaging has been applied to the diagnosis of acute ischemic stroke and achieved some results. Spiral CT perfusion imaging plays an auxiliary role in the early diagnosis of cerebral nervous system diseases, has an obvious effect on the identification of abnormal perfusion areas, and identifies the brain tissue of ischemic penumbra, which provides a clear direction for clinical treatment, that is, thrombolytic therapy, rescues the brain tissue of ischemic penumbra, and improves the prognosis of neurological function of brain injury. At present, the correlation between RBP4 and the expression level of RBP4 in patients with acute ischemic stroke has not been reported. This study analyzed the expression of RBP4 in patients with acute ischemic stroke to prove the correlation between them.

RBP4 (RBP4) is a transporter synthesized by liver and adipose tissue. It is mainly used for the transport and distribution of vitamin A in blood, most of which are distributed in the blood and cerebrospinal fluid.

Studies have shown that RBP4 is not only associated with obesity and diabetes but also causes risk factors for cardiovascular and cerebrovascular diseases such as metabolic syndrome, atherosclerosis, and coronary heart disease.

In addition, after thrombolysis, it can improve some brain circulation, correct some brain functions in time, and avoid some physical symptoms caused by large-area cerebral infarction.

## 2. Literature Review

The early diagnosis method of AIS is generally through brain CT examination. Through CT examination, we can intuitively understand the internal situation of the brain, so as to diagnose the disease, formulate a reasonable treatment plan, intervene in the patients, and improve their health [1]. AIS patients have many sequelae, which affect the body, language, and self-care ability of patients. Although they do not die, they bring serious physical and mental pain to patients. This paper analyzes the risk factors involved in intracerebral hemorrhage after thrombolysis in AIS patients. Through experimental comparison, it is finally concluded that intracerebral hemorrhage after thrombolysis in AIS patients will have the risk of systolic blood pressure and hyperlipidemia, and corresponding measures should be taken for these risks [1].

The disease has high incidence rate and high disability rate and brings economic burden to the patients. If the prognosis is not good, it will not only affect the quality of life but also need a lasting rehabilitation training, so that the whole family of the patient will fall into exhaustion. Wang et al. [2] found the relationship between serum retinol binding protein 4 (RBP4) and 8-isoprostaglandin (8-iso-pgf2) in patients with AIS and found that the level is related to the progress of the disease and has an impact on the patient's ability to live in the recovery period [2]. Zhang et al. [3] made some assumptions about the correlation between the serum retinol binding protein 4 level and the short-term outcome in patients with acute ischemic stroke. They selected AIS patients from a tertiary hospital for clinical comparative experiment. Finally, it is concluded that the higher the level of RBP4 in the serum of AIS patients, the better the short-term prognosis [3]. At present, in the study of Huang et al. [4], China's research on the pathogenesis of AIS shows that the onset of the disease is related to living habits and personal physique. In the intervention treatment after the disease, it is found that 4 (RBP4) is related to the prognosis of the disease. This paper studies and analyzes the correlation between the level of 4 (RBP4) in AIS patients and their prognosis. The higher the level of RBP4 in AIS patients, the lighter the symptoms after onset, and the better the prognosis [4].

Some studies have shown that serum RBP4 can promote macrovascular disease, which is related to atherosclerosis and can be used to predict clinical cardiovascular disease.

## 3. Data and Methods

### 3.1. Research Object

The first AIS patients in the Department of Neurology of our hospital were selected as the observation group. A total of 200 patients were treated from January 2020 to June 2021. At the same time, 100 healthy people were included as the blank group. All selected objects need to sign the informed consent form and have the right to know the contents of the study.

### 3.2. Inclusion Criteria

Firstly, the diagnostic criteria of Western medicine for AIS patients should be met, and the results of brain CT or MRI should be consistent with the symptoms of cerebral infarction. Secondly, timely medical examination should be sought after the onset of the disease, and the standards of hospitalization should be met.

Except for patients with other diseases, such as patients with malignant tumors or serious pathological changes of other organs, patients with cardiovascular and cerebrovascular diseases receiving thrombolytic therapy, patients with intracranial infection, patients with mental disorders and unconscious cognition, patients with incomplete clinical data, and patients who refused to cooperate or are not suitable to participate in this study for other reasons, all patients participating in this study have the right to know.

### 3.3. Grouping Method

Reference group: ECT screening and MRI angiography were used to determine the space occupying enhancement in the brain, and MRA angiography was used to determine the cerebral vascular obstruction, strengthen the monitoring of the state of the patient's brain tissue, and distinguish the brain tissue in the ischemic penumbra as an auxiliary treatment for clinical treatment. At the same time, the expression of 4 (RBP4) in patients was monitored, and the degree of brain injury was evaluated.

Observation group: all patients underwent spiral CT plain scan and perfusion scan in time after hospitalization. The perfusion scanning image was analyzed by software to obtain the TDC of the patient. At the same time, the expression of 4 (RBP4) in patients was monitored, and the degree of brain injury was evaluated.

Blank group: 100 healthy people were selected and their brain tissue was monitored and compared with the brain tissue of AIS patients, and the expression of 4 (RBP4) was monitored in healthy people.

### 3.4. Statistical Methods

In order to verify the role of the above 4 (RBP4) levels in AIS patients, the *R*^2^ value was obtained by the linear regression method under SPSS, and the *T* value and *P* value were obtained by the bivariate *t*-test.

The statistical method of *R*^2^ value is the ratio of regression residual to mean residual, as shown in the following formula:

(1) $$\begin{array}{c} R^{2}=\frac{\sum_{i}\left(x_{i}-\bar{x}\right)}{\sum_{i}\left(x_{i}-{\tilde{x}}_{i}\right)},\bar{x}=\frac{1}{n}\overset{n}{\underset{i=1}{\sum }}x_{i}. \end{array}$$

Among them, $\bar{x}$ is to investigate the arithmetic mean of sample sequence; ${\tilde{x}}_{i}$ is the ith regression value in the series; *x*_*i*_ is the ith input value in the sequence; *n* is the number of investigation samples.

The calculation algorithm of *T* value is shown in the following equation:

(2) $$\begin{array}{c} t_{\text{Value}}=\frac{\bar{x}-\mu }{\left(\sigma_{x}/\sqrt{n-1}\right)},\;\bar{x},\mu =\frac{1}{n,m}\sum_{i=1}^{n,m}x_{i},\sigma_{x}=\frac{1}{n-1}\sqrt{\sum_{i=1}^{n}{\left(x_{i}-\bar{x}\right)}^{2}}, \end{array}$$

where $\bar{x}$ is the mean value; *μ*  is the reference mean value; *n* is the sample maximum subscript; *m* is the maximum subscript of reference sample; and *σ*_*x*_ is the sample standard deviation.

## 4. Results

### 4.1. Routine Indexes and Detection Results of the Retinol Binding Protein 4 (RBP4) Expression Level of Patients before and after Treatment

#### 4.1.1. Comparison of Routine Index Test Data of Patients before and after Treatment

In this study, blood samples from patients with ARS and healthy people were collected, and the contents of total cholesterol (TC), triacylglycerol (TG), high-density lipoprotein cholesterol (HDL-C), and low-density lipoprotein cholesterol (LDL-C) were measured by using the automatic biochemical analyzer to obtain the data in Table 1.

In Table 1, compared with healthy people, the test results of TC and TG in patients with ARS after intervention in different examination methods and routine treatment were not statistically significant. This showed that the content of TC and TG in the body will not change greatly whether the patient is ill or not, which also showed that it is impossible to judge whether the patient has acute ischemic stroke and whether the condition has improved from the changes of total cholesterol and triacylglycerol.  Figure 1 is made according to the data in Table 1, which can facilitate readers to more clearly compare the differences between the two groups of data.

It can be clearly seen from Figure 1 that the expression levels of total cholesterol and triacylglycerol in ARS patients in the same group before treatment and after treatment were not statistically significant, and there was no statistical significance in the comparison of patients in different groups, Studies have shown that the expression levels of total cholesterol and triacylglycerol do not affect the severity of ARS patients.

The test data of high-density lipoprotein cholesterol and low-density lipoprotein cholesterol in different groups were statistically analyzed, as shown in Table 2.

In Table 2, compared with the healthy population, the comparison of HDL-C and LDL-C test data between the two groups before treatment and after treatment had no statistical significance. By comparing the test data of HDL-C and LDL-C of the two groups of patients with different examination methods and intervention, it was found that the data comparison of HDL-C and LDL-C of the two groups of patients was not statistically significant, and there was no significant difference between the data comparison of HDL-C and LDL-C of the same group of patients before and after treatment. This showed that the role of the disease in patients with ARS cannot be judged from the expression levels of HDL-C and LDL-C whether they are ill or not, and the expression levels of HDL-C and LDL-C in their bodies were not affected.  Figure 2 is obtained according to the data in Table 2.

It can be seen from Figure 2 that no matter what kind of examination method was used to intervene in ARS patients, there was no significant change in the expression levels of HDL-C and LDL-C in ARS patients after routine treatment, which showed that the disease development and prognosis of ARS patients cannot be judged by detecting the changes in the expression levels of HDL-C and LDL-C in ARS patients.

#### 4.1.2. Comparison of RBP4 Test Data before and after Treatment

After different imaging examination methods and routine treatment, ARS patients participating in this trial were compared and analyzed by detecting the expression level of retinol binding protein 4 before and after treatment by enzyme-linked immunosorbent assay (ELISA), and the correlation between CT perfusion imaging and patient prognosis was obtained as shown in Table 3.

In Table 3, compared with the healthy population, the RBP4 test results of ARS patients were lower, and compared with the RBP4 test data of the two groups of ARS patients before and after treatment, it can be seen that the content of RBP4 test data of ARS patients after routine treatment and after CT perfusion imaging was significantly higher than that of ARS patients in the reference group, and it can be found that compared with ARS patients in the same group, whether before or after treatment, the changes in RBP4 detection data in patients with ARS were also obvious, which also showed that the prognosis of patients can be reflected by detecting the changes of RBP4 in patients with ARS. Then, Figure 3 is obtained according to the data in Table 3.

In Figure 3, there was no significant difference in the expression level of RBP4 between the two groups of ARS patients before treatment. The changes of RBP4 expression level after treatment were different in patients with different examination methods. The expression level of RBP4 in patients in the observation group was higher after treatment.

### 4.2. Evaluation Results of NIHSS Score Scale, BI Score Scale, and MRS Score Scale of ARS Patients before and after Treatment

Through the NIHSS, BI, and MRS evaluation results of ARS patients before and after treatment as the evaluation indicators of clinical neurological deficit, ADL, and prognosis dysfunction, the correlation between RBP4 and CT perfusion imaging and the prognosis of ARS patients was analyzed and clarified, so as to provide convenient and fast detection indexes for the judgment of clinical treatment prognosis of ARS patients to improve the prognosis and treatment effect of patients with ARS.

The NIHSS score scale was used as an evaluation tool for the clinical judgment of patients' neurological deficit. The specific score range was 0–42 points. The higher the score, the more serious the patient's neurological deficit. Generally, 0-1 points were normal; 1–4: mild; 5–15: moderate; 15–20: moderate to severe; 21–42: severe. The specific evaluation results of different patients are shown in Table 4.

In Table 4, the NIHSS score results of the two groups before treatment are basically the same. The patients detected by CT perfusion imaging have a better prognosis effect, the neurological deficit has been controlled to a certain extent, and the short-term recovery is relatively optimistic, while the patients detected by traditional CT imaging have a relatively poor prognosis effect, there are generally moderate neurological deficits, and the short-term recovery was not as good as that detected by CT perfusion imaging.

The Barthel index refers to the measurement of the functional state of patients' activities of daily living. The individual score depends on the measurement of a series of independent behaviors. The total score ranges from 0 to 100. The scoring criteria are as follows: more than 60 points for those with only mild disability but basic life management; 40–60 points for those with moderate disability who need help in life; 20–40 points for those with severe disability who need great help in life; less than 20 points for those who are completely disabled and completely dependent on life. Since the late 1980s, this assessment method has also been widely used in the assessment of activities of daily living in China. The scoring results of different groups of patients are shown in Table 5.

In Table 5, the patients in the two groups were severely disabled and needed the help of others before treatment. After clinical treatment, the BI score of the observation group was significantly higher than that of the reference group, and the short-term recovery effect was good to realize self-care.

MRS was used to measure the recovery of neurological function in patients with ARS. There were 6 specific scoring levels. The specific scoring standard was as follows: 0 for complete asymptomatic; despite symptoms, there was no obvious disability; 1 point for being able to complete all frequently engaged responsibilities and activities—mild disability; 2 points for those who cannot complete all the activities they can engage in before, but can handle personal affairs without help—moderate disability; 3 points for those who need some assistance but do not need assistance in walking—severe disability; 4 points for those who cannot walk without the assistance of others and cannot take care of their own physical needs—severe disability; 5 points for those who are bedridden, incontinent, and need continuous nursing and care; death rate was 6 points. The scores of different groups of patients were statistically analyzed to obtain the data in Table 6.

In Table 6, the MRS scores of the two groups of patients before treatment are not very ideal. They need their assistance to complete the action function, which belongs to severe disability. After the clinical intervention, the MRS scores of the observation group were significantly higher than those of the reference group, and the short-term treatment effect was obvious, so they can walk independently.

## 5. Discussion

For stroke caused by cerebral ischemia or injury, fibrin can be used for vascular thrombolysis. Fibrinolytic system is closely related to ischemic cerebrovascular disease. The brain nerve is complex, and the effective treatment time is less than 3 hours. If we do not timely understand the type of disease and brain tissue injury, there will be serious consequences. The images of spiral CT plain scan and perfusion imaging provide doctors with brain morphology scanning and the status of lesions can be judged through CT imaging. Compared with the previous coarse screening of ECT, spiral CT plain scan, and perfusion scan, MRI angiography determines the space occupying in the brain, and MRA angiography can identify the lesions of patients more comprehensively, so as to make more accurate judgment and give the best treatment plan.

Song et al. [5] showed that the expression of brachial index combined with 4 (RBP4) and lipoprotein phospholipase A2 could predict the development of diabetic patients with ischemic stroke [5]. Hou et al. [6] also showed that 4 (RBP4) can predict the disease progress of AIS patients and reflect the size of the brain tissue damage area of patients [6]. In the study of Fan et al. [7], based on the ultra-wide angle fluorescein angiography (VDV) image for diabetic retinopathy staging, a multimodal deep learning model was mentioned. The images generated by the ultra-wide fluorescein angiography showed that all the lesions were removed, while the normal vascular structure was preserved. The difference in image directly reveals the distribution of biomarkers. The thermal icon shows the leakage area, and the location is basically consistent with the lesion area in the original image [7]. Cheng [8] studied the relationship between monocyte/HDL cholesterol ratio, cerebral collateral circulation, and neurological deficit in patients with acute ischemic stroke (AIS). It can be concluded that MHR, cerebral collateral circulation, and neurological deficit can effectively reflect the inflammatory response and blood flow compensation ability of AIS patients and have certain guiding significance and value in predicting the neurological deficit of AIS patients [8].

All subjects have signed the informed consent form, all examination results and patients' privacy have been protected, and the samples or relevant medical data collected from the patients will be marked with the study code instead of the patient's name. Without violating the confidentiality principle and relevant laws and regulations, only the personnel participating in the study can access the basic clinical data of patients.

## 6. Summary

This study explored the correlation between the expression level of RBP4 and CT perfusion imaging and prognosis of AIS patients through grouping experiments and different examination methods for different groups of patients. According to the above data, AIS patients were treated with routine treatment after CT perfusion imaging. Only the expression level of RBP4 changed before and after treatment, and the expression of RBP4 increased with the appearance of treatment effect, that is, the expression level of RBP4 was correlated with CT perfusion imaging and the prognosis of AIS patients. It can provide convenient and fast detection indicators for the prognosis judgment of AIS clinical treatment, improve the prognosis and treatment effect of patients, pay attention to details, take the benefit of patients as the prognosis judgment, and improve the quality of life of patients.

## Figures and Tables

**Figure 1:** Comparison of total cholesterol and triglyceride data in different groups before and after treatment.

**Figure 2:** Comparison of HDL-C and LDL-C test data in patients with ARS.

**Figure 3:** Comparison of RBP4 expression levels in different groups before and after treatment.

**Table 1:** Comparison of total cholesterol and triacylglycerol data in different groups before and after treatment.

Grouping	Total cholesterol			Triacylglycerol		
	Before treatment	After treatment		Before treatment	After treatment	
		Day 7	Day 14		Day 7	Day 14
Observation group	4.28 ± 1.08	4.37 ± 0.93	4.48 ± 1.07	1.14 ± 0.21	1.16 ± 0.13	1.15 ± 0.14
Reference group	4.29 ± 1.23	4.40 ± 1.03	4.47 ± 1.13	1.13 ± 0.23	1.14 ± 0.15	1.16 ± 0.18
Blank group	4.35 ± 1.35			1.23 ± 0.35		

**Table 2:** Comparison of the HDL-C and LDL-C test data in patients with ARS (the data are from the basic clinical data of patients in our hospital).

Grouping	HDL-C			LDL-C		
	Before treatment	After treatment		Before treatment	After treatment	
		Day 7	Day14		Day 7	Day14
Observation group	1.06 ± 0.26	1.05 ± 0.25	1.07 ± 0.23	2.64 ± 0.88	2.71 ± 0.67	2.73 ± 0.54
Reference group	1.04 ± 0.31	1.06 ± 0.36	1.05 ± 0.34	2.66 ± 0.84	2.73 ± 0.69	2.73 ± 0.61
Blank group	1.05 ± 0.26			2.71 ± 0.72		

**Table 3:** Comparison of RBP4 expression levels in different groups before and after treatment (the data are from the basic clinical data of patients in our hospital).

Grouping	*N*	Before treatment	After treatment	
			Day 7	Day 14
Observation group	100	21.36 ± 5.34	33.13 ± 4.53	39.84 ± 4.68
Reference group	100	20.67 ± 4.68	27.51 ± 4.67	33.94 ± 3.87
Blank group	100	45.84 ± 2.16		

**Table 4:** Comparison of the NIHSS scores in different groups (the data are from the basic clinical data of patients in our hospital).

Grouping	*N*	Before treatment	After treatment	
			Day 7	Day 14
Observation group	100	17.35 ± 3.15	11.51 ± 2.37	4.28 ± 1.28
Reference group	100	16.57 ± 4.58	13.29 ± 3.21	7.18 ± 2.17
Blank group	100	0		

**Table 5:** Comparison of BI scores of patients in different groups (the data are from the basic clinical data of patients in our hospital).

Grouping	*N*	Before treatment	After treatment	
			Day 7	Day 14
Observation group	100	43.59 ± 5.59	59.28 ± 5.46	86.18 ± 4.26
Reference group	100	41.17 ± 6.15	50.03 ± 6.24	72.73 ± 3.29
Blank group	100	100		

**Table 6:** Comparison of the MRS scores in different groups (the data are from the basic clinical data of patients in our hospital).

Grouping	*N*	Before treatment	After treatment	
			Day 7	Day 14
Observation group	100	3.94 ± 3.25	2.05 ± 2.31	1.31 ± 1.01
Reference group	100	3.95 ± 4.34	2.61 ± 3.14	2.03 ± 2.61
Blank group	100	0		

## Data Availability

The data underlying the results presented in the study are available within the manuscript.
